The article "An Image Processing Approach for Detection of Prenatal Heart Disease" was retracted in 2023. Reasons: signs of a paper mill; compromised peer review; unreliable results or conclusions.

# An Image Processing Approach for Detection of Prenatal Heart Disease

**DOI:** 10.1155/2022/2003184

**Published:** 2022-08-02

**Authors:** Saravana Selvan, S. John Justin Thangaraj, J. Samson Isaac, T. Benil, K. Muthulakshmi, Hesham S. Almoallim, Sulaiman Ali Alharbi, R. R. Kumar, Sojan Palukaran Thimothy

**Affiliations:** ^1^Faculty of Engineering & Computer Technology, AIMST University, Bedong, Kedah 08100, Malaysia; ^2^Department of Computer Science Engineering, Saveetha School of Engineering, Saveetha Institute of Medical and Technical Sciences (SIMATS), Chennai, Tamil Nadu 600124, India; ^3^Department of Biomedical Engineering, Karunya Institute of Technology and Sciences, Coimbatore, Tamil Nadu 641114, India; ^4^Department of Information Technology, M.Kumarasamy College of Engineering, Karur, Tamil Nadu 639113, India; ^5^Department of Information Technology, Panimalar Engineering College, Chennai, Tamil Nadu 600123, India; ^6^Department of Oral and Maxillofacial Surgery, College of Dentistry, King Saud University, PO Box-60169, Riyadh-11545, Saudi Arabia; ^7^Department of Botany and Microbiology, College of Science, King Saud University, PO Box-2455, Riyadh-11451, Saudi Arabia; ^8^Department of Civil Engineering, University of Houston, Texas, USA; ^9^Faculty of Mechanical Engineering, Arba Minch Institute of Technology (AMIT) Arba Minch University, Ethiopia

## Abstract

Prenatal heart disease, generally known as cardiac problems (CHDs), is a group of ailments that damage the heartbeat and has recently now become top deaths worldwide. It connects a plethora of cardiovascular diseases risks to the urgent in need of accurate, trustworthy, and effective approaches for early recognition. Data preprocessing is a common method for evaluating big quantities of information in the medical business. To help clinicians forecast heart problems, investigators utilize a range of data mining algorithms to examine enormous volumes of intricate medical information. The system is predicated on classification models such as NB, KNN, DT, and RF algorithms, so it includes a variety of cardiac disease-related variables. It takes do with an entire dataset from the medical research database of patients with heart disease. The set has 300 instances and 75 attributes. Considering their relevance in establishing the usefulness of alternate approaches, only 15 of the 75 criteria are examined. The purpose of this research is to predict whether or not a person will develop cardiovascular disease. According to the statistics, naïve Bayes classifier has the highest overall accuracy.

## 1. Introduction

Congenital heart disease (CHD) is predicted to affect 8.7 out of 2000 liveborn newborns. In the industrialized countries, congenital abnormalities are among the major causes of newborn death, with serious CHD accounting for more fatalities than any other kind of deformity [1]. Fetal echocardiogram is one of the prenatal exams that may be done in the first stage. The cardiovascular screening test, on the other hand, is best conducted around 18 and 22 weeks of pregnancy, and so many anatomical features may still be seen well beyond that. If a prenatal diagnosis of fetal CHD is made, pregnant women are sent to a tertiary medical center that can provide an accurate prenatal testing, specialist neonatal intensive care, delivery planning, and emergency cardiac surgeries to assist the fetus survive. Over the last decade, coronary artery disease, often known as coronary heart disease, has been the top cause of death worldwide [2]. According to the WHO, over 18 million annual deaths every year as a cause of heart illness, including coronary heart disease and intellectual stroke, accounted for 82 percent of these deaths. Large numbers of deaths are common in rural countries [3] personally and professionally actions, as well as inherited vulnerability, all have a role in the development of heart disease. Alcohol, liquor, and cigarette use, as well as stress and lack of physical activity and physiology such as obesity, are all key risk factors.

The article "An Image Processing Approach for Detection of Prenatal Heart Disease" was retracted in 2023. Reasons: signs of a paper mill; compromised peer review; unreliable results or conclusions.

The detection of a congenital abnormality before birth provides a unique circumstance. Prenatal diagnosis lowered the probability of mortality with planned heart surgery for babies who did not have extra risk factors and whose families sought care. However, due to a lack of understanding about the condition and its unclear prognosis, pregnant women who learn about prenatal CHD suffer tremendous sadness, rage, loss of attachment for the fetus, and concern [4]. A large percentage of women have been found to have stressful symptoms, with approximately 40% above clinical threshold levels for posttraumatic stress disorder. Furthermore, the parents may criticize or feel responsible for each other, resulting in a rift among them. Pregnant women seek advice from a number of healthcare providers during this trying time to learn more about the condition [5]. Counseling from healthcare providers has been shown to have a significant impact on judgment, and clinicians' specific roles, such as empathizing with parents' feelings, trying to coordinate with other medical practitioners on their behalf, and continuing to support parents' decisions, have also been noted. To deliver superior healthcare, health providers must fully comprehend the experience of people with fetal CHD, the illness, and its therapy trajectory [6].

The article "An Image Processing Approach for Detection of Prenatal Heart Disease" was retracted in 2023. Reasons: signs of a paper mill; compromised peer review; unreliable results or conclusions.

These days, the amount of data generated in the last few years exceeds that of the whole human race's history. As a result, the need of the hour is to identify the best methods for dealing with these vast amounts of data. Intelligence bioinspired algorithms are used to solve issues that are dynamical and contain partial and faulty data. Because they can absorb and modify like biological beings, these algorithms are referred to as intelligent [7]. However, because of the quick advancement of this discipline, the bulk of bioinspired algorithms have been overlooked. Some of the most well-known past studies in the topic of organic algorithms were reviewed. To address a confined optimization issue, the image processing proposes a shrinking coefficient to see if the particles are in a viable zone. They focused their study on the subject of protein structure and function structure prediction. Healthcare experts developed their own method for multimodal issues by studying how plants grow [8]. They chose the issue of specific proteins structure prediction and termed it image processing. It is used to estimate the structure and movement off heart function.

Heart disease has caused scientists a tremendous deal of concern. Determining the presence of the ailment within a person is among the most challenging components of heart disease treatment. Medical authorities were not really better at determining heart disease, and initial techniques were not particularly good at finding it. A wide range of medical devices is commercially available for predicting heart illness. They have two major flaws: one is that these are prohibitively expensive, and the second is that they may have failed to effectively predict the risk of cardiovascular disease in people. Only 68 percent of medical experts could correctly predict heart illness, as shown in a recent WHO questionnaire [9]. As a result, there is a sizable scientific community focused in predicting heart disease in people. Advanced scientific incorporation has finally opened a plethora of new opportunities in an array of sectors, including drug research. Microscope to maritime engineering is all examples of machine learning applications. Some of the most essential computer science approaches have also been used in clinical research; machine learning has gained in terms of popularity as computing capabilities have expanded. AI is a technology that is widely employed in a variety of areas because it does not includes a single algorithms for different datasets [10]. The programmable features of machine learning add a lot of power and bring up new opportunities in industries like medical science.

Since many years, machine diagnostic systems were used. Clinical diagnosis is well recognized to be objective, relying not only on available facts but also on the surgeon's experience. Computerized translation has been proposed as major contributor for analyzing the physician's interpretations. Due of its high capability of detecting complicated correlations in large datasets, machine learning algorithms are increasingly being used to build CAD systems [11]. The large volume of medical information necessitates some useful classification algorithms to aid in data analysis. The accuracy of categorization algorithms employed in disease diagnosis is unquestionably a critical factor to consider. The majority of medical research results has a higher-dimensional feature dataset. In order to remove extraneous elements from a data source, image compression is crucial in diagnostic systems. The feature reduction process can help reduce dataset complexity while also improving performance of the classifier. Screening tests become faster, more convenient, and less expensive when the number of unnecessary characteristics in the model is reduced [12]. The current study is aimed at finding the favorite asset subset for a lymphography database in order to increase diagnostic performance. A trade-off must be made between computing time and the accuracy of the provided relevant feature alternatives.

The article "An Image Processing Approach for Detection of Prenatal Heart Disease" was retracted in 2023. Reasons: signs of a paper mill; compromised peer review; unreliable results or conclusions.

Because it incorporates so many factors and is so complicated, cardiovascular disease is among the most challenging illnesses to forecast in medical research. Since this tool uses feature maps and their multiple data kinds under various situation for heart disease prediction, postprocessing may be the greatest option for achieving maximum predictive accuracy not only heart problems but also many other infections. To forecast the risk of cardiovascular illness, techniques such as NBB, KNN image processing, and KNN are employed. Every algorithm has a niche; for example, naive Bayes predicts heart disease using probability. To create predictions regarding new patients, all of these approaches rely on previous patient information. To create predictions regarding new patients, all of these approaches rely on previous patient information. This heart disease prediction system assists doctors in early detection of heart disease, ultimately saving lives. This review article [13] examines a wide range of machine learning approaches in the field of heart disease. The survey article's last portion will evaluate and contrast many machine learning methods for heart disease on various factors. It also shows how machine learning techniques might be used to treat heart illness in the future. This study also looks at how deep learning may be used to predict cardiac disease.

The article "An Image Processing Approach for Detection of Prenatal Heart Disease" was retracted in 2023. Reasons: signs of a paper mill; compromised peer review; unreliable results or conclusions.

Humans in this fast-paced entire globe would like to survive a very wealthy lifestyle, so those who work like machines in order to obtain a great deal of money and live quite comfortably. As an outcome, they neglect the importance of their self, as well as their food preferences and a whole lifestyles change over the course. Those who seem to be more strained [14] have cardiac problems and other health issues at an early age, and they do not even consider giving themselves sufficient sleep and eat whatever they can get. It is a universal truth that the heart is the most important organ in the human body, and that if it is harmed, it will influence the rest of the body's other organs. As a result, it is critical for patients to get a heart disease diagnosis. Individuals seek the advice of healthcare professionals, although their predictions are not always right. Quality service includes appropriately diagnosing patients and providing effective therapies. Poor clinical judgments can have devastating effects, which is unacceptably dangerous. Clinical testing must also be kept to a minimum in hospitals. They can attain these outcomes by utilizing relevant machine information and decision-making technologies [15].

The healthcare sector generates enormous amounts of data, which is sadly not “collected” for additional information that could help decision-makers make better choices. Often, hidden patterns and connections go unnoticed. Improved data mining methods may be able to help with this problem [16]. This study builts a prototype Heart Disease Prediction System using data mining approaches such as DT, NB, and NN (HDPS). The findings show that each technique has a different advantage in accomplishing the stated mining targets' aims and objectives. Standard decision support systems will not be answering complicated what-if questions, but HDPS can. In this paper, prenatal heart disease is detected by [17] naive Bayes classifier using machine learning approach and Bayesian interpretation principles. Naive Bayes classifier is used for automated disease detection and development. It is effectively detecting a heart disease background with less training data. In Section 1, the overall introduction about the prenatal heart disease is explained, and this prediction method and related work explain various methods used in heart disease detection and this defects in Section 2. The proposed methodology is described in Section 3, and detailed results and discussion are mentioned in Sections 4 and 5, followed by conclusion in Section 6.

## 2. Related Works

Many outstanding researches were already done in the field of illness predictions utilizing machine learning technique, with a focus on machine learning in clinical labs. Various algorithms are used to detect heart disease. Multiple linear regression is effective for estimating the risk of coronary heart disease, according to the model. The research is based on a raw data collection of 2000 instances with 20 different features that were previously established [10]. The data is divided into two parts, with 70% of the material being used to train the machine and 40% being utilized for testing reasons. As can be seen from the results, the consequence of the recreation algorithms is the best in compared to other algorithms. WEKA software was used to create a projection framework for cardiac illnesses utilizing SMO, KStar, Bayes Net, j48, and Multilayer perception. Using *k*-fold validation, J48 procedures and multilayered perception outperform KStar regarding the results from single variable SMO and Bayes Net mainly on processes that can detect chronic illness using naive Bayes, artificial neural network (ANN), support vector machine (SVM), and decision tree, to retrieve the data center, precision in the outcomes. A comparison examination of classifiers is done in order to discover the right output at a specific scale. This experiment yielded the best SVM precision, with naive Bayes assisting the low accuracy in findings.

The article "An Image Processing Approach for Detection of Prenatal Heart Disease" was retracted in 2023. Reasons: signs of a paper mill; compromised peer review; unreliable results or conclusions.

Nonlinear classification methods are being used to forecast cardiac disease. Widedata techniques like HDFS and map reduction with SVM are suggested for prediction of heart disease with an optimum set of characteristics. The use of different data mining algorithms to discover cardiac disease was also examined in this study. HDFS to store large amounts of data over several nodes, as well as employing SVM to perform the prediction algorithm across multiple nodes. It is utilized in a similar way, with faster processing times than typical. One of the most often used data categorization approaches is linear discriminant analysis (LDA). The complete set of characteristics that best differentiates two classes of object is found using LDA. The generated mixtures can be used to create a linear classifier [18]. In each given dataset, this approach increases the ratio of between-class variation within each variance, ensuring maximum reparability. In this work, cross-validation was used to maximize the number of PCs used in developing the LDA model. The best number of PCs was determined by cross-validation using the greatest discrimination rates. When 10 PCs were used, the best LDA model was created, with discrimination rates of 94.8 percent and 89.4 percent in the testing and projection sets, accordingly. Nonlinear classifiers are frequently less effective than linear classifiers when an issue is nonlinear and the classification borders cannot be estimated accurately with linear separating hyperplane. If the issue is linear, a simplified linear classifier should be used.

The article "An Image Processing Approach for Detection of Prenatal Heart Disease" was retracted in 2023. Reasons: signs of a paper mill; compromised peer review; unreliable results or conclusions.

Among the most widely used data mining approaches is the decision tree. However, the majority of studies have used the J4.8 decision tree, which is based on the performance gain and binary differencing. Other effective versions of decision trees include the Gini index and gain ratio, which are less commonly utilized in the detection of heart disease. Also known to yield more effective decision trees are alternative discretization approaches, voting methods, and decreased error trimming. This study looks into using a variety of approached by [19] to improve the effectiveness of several types of decision trees in the detection of heart disease. This study makes use of a commonly utilized benchmark data collection. The sensibility, selectivity, and accuracy of the various decision trees are determined to assess their performance. Because the decision tree is among the data mining methods that cannot directly manage statistical parameters, the continuous characteristics must be discretized. For prolonged features, the C4.5 and J4.8 decision trees employ binary fuzzification. Cross-discretization approaches, on the other hand, have been shown to create accurate classification trees than binary discretization, although they are less commonly utilized in heart disease detection studies. Using hybrid classification voting and decreased error trimming to improve accuracy of decision tree in the detection of patients with heart disease is another key improvement. More complicated models should, on the surface, yield more precise findings.

Various medical decision support methods are described by [20] in this respect, and past work has used a variety of medical criteria and risk variables, as well as various data mining approaches. The degree of accuracy stated in each of those articles is defined by the amount of parameters used and the data mining used. However, the number of variables and datasets used in the studies was insufficient to claim great precision. Using 14 characteristics and the *K*-nearest neighbor classifier, we were able to attain an accuracy of around 79%. Furthermore, a variety of popular classifiers were tested to demonstrate the superiority of the kNN classifier-based heart disease diagnosis. It is a major source of inspiration for our study. Following that, mining techniques are used. Using different data mining techniques, data mining is the process of extracting information from a stored database in order to obtain the hidden answers to your queries. The Information Retrieval Database Process is another name for this procedure. To get understanding, the KDD Process includes the processes of data selection, data preparation, data transformation, and data mining techniques. This information may then be used by healthcare professionals and clinicians to better forecast the condition.

The article "An Image Processing Approach for Detection of Prenatal Heart Disease" was retracted in 2023. Reasons: signs of a paper mill; compromised peer review; unreliable results or conclusions.

To predict heart illnesses, a random forest classifier (RFC) technique is developed by [21]. The first stage of the proposed model, which focuses on feature selection, is aimed at constructing various feature extraction methods for reducing dimensionality of the heart diseases dataset, including such optimization technique (GA), relief-*F*, principal component analysis (PCA), sequential forward floating search (SFFS), sequential backward floating search (SBFS), and Fisher. In the second phase, the resulting feature subsets are input into the RFC for effective classification, shifting from feature extraction to model creation. GA-RFC was reported to have the greatest accuracy rate of 87 percent. Using GA, the size of the original input area is decreased from eighteen to six elements. Lymph disease detection is a popular study topic in research. To identify multiclass issues such as dermatology, lymphography, and image segmentation datasets collected from the UCI (University of California Irvine) machine learning databases, a unique hybrid classification method that is based on C4.5 decision tree algorithm including one technique was developed. The C4.5 system was used to classify all of the samples in this study, and they obtained accuracy rate of 84.48 percent, 88.79 percent, and 80.11 percent for dermatological, segmentation techniques, and lymphography databases, accordingly, using classifiers. For the above databases, the proposed methodology predicated on C4.5 decision trees also one approach achieved 89 percent, 90 percent, and 87 percent, accordingly. For text categorization, including lymph disease datasets, decomposing approaches such as one-per-class (OpC), pairwise coupling (PWC), and error-correcting output codes (ECOC) were used. The comparison was done using three distinct methodologies for basic classifiers, including the multilayer perceptron (MLP) as a CNN architecture, the nearest neighbor (NN) as a binary classifier, and the support vector machine (SVM) as a kernel machine. Using OpC, PWC, and ECOC, the experimental outcomes for MLP were 82.90 percent, 79.32 percent, and 75.84 percent, respectively. These feature outcomes for the NN classifier were 78 percent, 75 percent, and 77 percent, respectively. Finally, SVM employing ECOC, PWC, and OpC yielded performance values of 88 percent, 80 percent, and 77 percent, respectively. Some of the most current classification performance for the cardiovascular disease dataset from various studies.

The article "An Image Processing Approach for Detection of Prenatal Heart Disease" was retracted in 2023. Reasons: signs of a paper mill; compromised peer review; unreliable results or conclusions.

Data mining and machine learning methods are analyzed by [1] which were used to detect cardiac disease. Techniques for machine learning have been shown to be useful in a number of actual data mining techniques. Professional versions of these methods, as well as effective interfaces to multiple databases and also well user interfaces are now available from dozens of firms across the world. However, these first-generation methods have serious drawbacks. They usually presume that the data only has numerical and symbolic properties and that there is no text, visual features, or raw sensor readings. They presume the information has been meticulously gathered into a single database for a data mining purpose [22]. A model for predicting cardiac disease using data mining technologies such as the naive Bayes classifier and the decision tree. The validation tests are used to forecast the classifier's efficiency. For the provided dataset, the decision tree outperforms the naive Bayes classifier, according to the research. The research evaluated the artificial neural networks (ANNs), decision tree, RIPPER classifier, and support vector machine to predict and diagnose heart diseases (SVM). Mining techniques was shown to be the least accurate of the four classifiers for disease prediction after rigorous testing. Furthermore, modern methods are frequently fully automated, obviating the requirement for knowledgeable users' input at important stages of data generalization search. The most important thing is to identify hidden patterns using data mining tools. The J48 techniques that use the UCI dataset have worse accuracy than the LMT methods.

The ANN data mining method [23] was used to detect heart problems. Because of the rising expense of diagnostics, a new technology was needed to forecast readily accessible and low-cost cardiac problems. The prediction technique is used after an estimate to determine the patient's state based on several restrictions such as blood pressure, heart rates, cholesterol, and pulse rate. In Java, the technology is well known for its accuracy. In healthcare, there seems to be an abundance of data, so there is no effective analytic tool to uncover hidden links in the data. There are several techniques and methods for generating new knowledge, ‘data mining' is a fast expanding one that is valuable for generating new details from big preexisting datasets, particularly in the medical profession. Every year, millions of death are a result of heart disease. The identification of cardiovascular disease appears to be a critical requirement of data mining tools. A doctor can diagnose heart disease by using data. The goal of this study is to compare different categorization approaches for heart disease diagnosis. “Data abundant but knowledge poor” is a well-known statement in the health sector. Humans are hopeful that data mining approaches will be able to assist as a remedy in this case. For a satisfactory outcome, many data mining approaches might be used. The purpose of this work is to provide facts on various parts of information utilizing data mining algorithms in order to take adequate safeguards against heart problems. The patient's activities are constantly monitored. Any act takes place. The clinician and patients are then educated on illness risk antonyms. Doctors can utilize machine learning techniques with the assistance of digital technology to detect cardiac illnesses at an early stage. This study gives you an idea of how data mining is used to predict cardiovascular illnesses. ANN is less predictive, and it is difficult to face problems on the network. ANN can work with numerical information, and this processing power depends on the structure of hardware.

The article "An Image Processing Approach for Detection of Prenatal Heart Disease" was retracted in 2023. Reasons: signs of a paper mill; compromised peer review; unreliable results or conclusions.

The development of a prediction system that would identify heart illness utilizing the child's medical information, as well as input parameters, was also considered. Following an assessment of the dataset's record, data screening and consolidation were carried out. Machine learning approaches are being used to forecast cardiac disease. The cardiac program uses two key goals when it comes to prediction. This software does not take into account any prior knowledge of the sets of data. Due to the large number of datasets, the devices used had to be scalar to run. Precise decision-making is useful to the medical professional because it results in 86 percent accuracy in evaluating and 88 percent accuracy in teaching. The sickness was assumed using data mining methods in this research. It contains an analysis of current methodologies for extracting information from the datasets, and it will be beneficial to healthcare professionals. The goal may be met by using consumption to create a scientific decision tree [24]. For categorization issues, the decision tree method is more effective. Building a tree and implementing the graph to the database are the two processes in this approach. CART, CHAID, ID3, J48 and C4.5 are examples of popular decision tree algorithms. The J48 method was used to create this systems. The J48 method uses a trimming process to build a tree. Scaling is a technique for lowering a massive tree volume by removing overfit data, which causes low predictive performance. The J48 approach recursively classifies data until it is categorized as correctly as possible. This approach has a lower level of accuracy on training data. The ultimate objective is to make a less adaptable and exact tree. Because graded training data differs so much from sampling training examples, this strategy does not generate adequate results.

The article "An Image Processing Approach for Detection of Prenatal Heart Disease" was retracted in 2023. Reasons: signs of a paper mill; compromised peer review; unreliable results or conclusions.

Neural fuzzy system (DNFS) [25] approaches for evaluating and forecasting various cardiac conditions are used. The research into the therapy of cardiac disease was examined in this publication. The major goal of this study is to develop a smart and low-cost system, as well as to improve the present system's efficiency. In this article, data mining methods are largely employed to enhance heart disease predictions. The SVM and neural networks show exceptionally promising outcomes in heart disease prediction, according to the findings of this study. Even data mining technologies are not promising when it comes to forecasting heart disease. A fuzzy decision analysis system based on an optimization technique for forecasting heart disease risk levels. The fuzzy decision support system (FDSS) that we have presented works like this: (i) collect and process the dataset, (ii) choose effective characteristics using various approaches, (iii) use GA to construct weighed fuzzy rules tied to specific attributes, (iv) construct the FDSS using obtained fuzzy knowledge base, and (v) prediction heart disease tests using real-world data reveal that the proposed creative technique is successful. Fuzzy logic is a subjective computational framework that is used to describe things in the real world that are inaccurate. The fuzzy logic system (FLS) is a decision making tool that is modelled after the fuzzy rule-based system (FRBS). The usage of DSSs in medical technology is on the rise these days. The decision support systems are used by the majority of systems which require a computer-aided system. Even though some institutions utilize DSSs, they are only capable of handling simple queries instead of more complicated ones. Clinical judgments are frequently made based on an expert's expertise and intuition, rather than the system's underlying patterns. As a result, the quality of service provided to patients is impacted. FRBS provides inaccurate data inputs. Fuzzy logic is not have systematic approach for solving problems.

For the detection of cardiac illness, a novel technique depending on the coactive neurofuzzy inference system (CANFIS) was described. [26] suggested CANFIS model combines the adaptive capacity of neural networks with the descriptive method of fuzzy logic, which merged with a genetic algorithm to identify the existence of the sickness. The CANFIS model's performance was measured both training and classification levels of accuracy, and the findings revealed that the suggested CANFIS model had a great potentiality in heart disease prediction. The CANFIS model combines adjustable fuzzy inputs with a flexible neural network to estimate complicated functions quickly and reliably. Because fuzzy inference algorithms combine the informative aspect of rules (MFs) with the capability of neural networks, they are also useful. When the basic function to represent is extremely variable or locally severe, these types of networks handle problems more effectively than neural networks. It has been demonstrated that GA is an effective strategy for autotuning CANFIS settings and selecting the best features and functionality. The reality is that algorithms cannot replace people, and clinicians may discover more about best methods for assessing regions that computer-aided detecting emphasizes by comparing results of software detecting with pathology discoveries. Cardiovascular Disease dataset from the UCI Machine Learning was examined, highly processed, and scrubbed out in order to prepare it for categorization. Coactive neurofuzzy modeling has been offered as a reliable and robust approach for identifying a nonlinear link and mapping across various characteristics.

The article "An Image Processing Approach for Detection of Prenatal Heart Disease" was retracted in 2023. Reasons: signs of a paper mill; compromised peer review; unreliable results or conclusions.

## 3. Proposed Methodology

### 3.1. Naive Bayes Classifier

A naive Bayes method is being used in the suggested system for detecting heart disease, with specifications such as thalassemia, age, sex, max heart rate, resting blood pressure, chest pain type, ST depression induced, serum cholesterol, resting ECG, fasting blood sugar, peak exercise ST, exercise-induced angina, and number of major vessels being considered [13]. In comparison to state-of-the-art approaches, the suggested technique allows patients to adjust without professional intervention while without reducing detection accuracy for uncommon abnormal classes. It begins by presenting a method for successfully familiarizing oneself with parametric patterns. Prior to the occurrence of cardiac arrhythmia, readers can quickly distinguish patterns between various data. Later on, it goes into how to detect parameter ranges that are out of the ordinary. Age and gender are two factors that might impact the irregular ranges of several measurements. Finally, the essay depicts the advancements made to increase predicting accuracy of the parameters. The formula for naive Bayes classifier is as shown in Equation (1). Averaging, controlling outliers, and using morphology identification algorithms are some of the methods used. The naive Bayesian categorization implies predictions independent and is predicated on Bayesian' theorem. The naive Bayesian system is easy to build but does not requires repetitive parameter estimation, making it appropriate for large datasets. The suggested machine learning method is depicted in Figure 1 in a simplified manner. The classification technique typically works brilliantly and is widely used, outperforming more sophisticated classification approaches due to its basic nature.

(1) $$\begin{array}{c} f\left(x_{i}\left|y\right.\right)=\frac{f\left(y\left|x_{i}\right.\right)f\left(x_{i}\right)}{f\left(y\right)}, \end{array}$$

where *f*(*x*_*i*_|*y*) is a probability of instant *y* in class of *x*_*i*_ and *f*(*y*|*x*_*i*_) is a probability of generating instant *y* in class of *x*_*i*_. *f*(*x*_*i*_) is a probability occurrence of class *x*_*i*_ and *f*(*y*)is the instance of*y*occurring. Our approach is based on establishing a patient-specific baseline for the suggested deviation assessment, which is designed to detect modest deviations in sign structure from its usual state towards any of the irregularity classifications. Our approach is based on the idea that the individual signal highlights for various abnormal breakdowns produced by edge-based deviation inquiry. We suggest a unique guided nonlinear shift to restructure the signs geometries into symmetrical depiction in the component space to address the heart disease.

The article "An Image Processing Approach for Detection of Prenatal Heart Disease" was retracted in 2023. Reasons: signs of a paper mill; compromised peer review; unreliable results or conclusions.

### 3.2. Bayes Theorem

Bayes' theorem, often referred as Bayes' rule, Bayesian reasoning or Bayes' law, is a mathematical formula for calculating the probabilities of an occurrence based on ambiguous information [27]. It connects the conditionally and terminal possibilities of two random occurrences in Bayesian inference.  Figure 2 shows the working principle of naïve Bayes classifier. Bayes theorem contains several probabilities which combine into one effect (M). Several independent variables are defined (*x*_*i*_, *i* = 0, 1, 2, 3 ⋯ .*n*_*x*_). Equation (2) derives the Bayes theorem. Assuming initial instant probability is*f*(*x*_*i*_), conditional possibilities of*i*^*th*^class produce one effect is*f*(*x*_*i*_|*y*).

(2) $$\begin{array}{c} f\left(x_{i}\left|M\right.\right)=\frac{f\left(M\left|x_{i}\right.\right)f\left(x_{i}\right)}{\sum_{i=1}^{p_{c}}\left(M\left|x_{i}\right.\right)f\left(x_{i}\right)}. \end{array}$$

This may be expressed as follows: if we witness a specific incident (effect), the chance that it was caused by the *i*^th^ causes is related to the cause's possibility twice the cause's probability of producing the effect. The *f*(*x*_*i*_|*M*) is clearly dependent on initial probabilities of the causes. This provides the appearance that the formula is sterile at first glance. In practice, the Bayes formula has the ability to enhance *f*(*x*_*i*_) knowing as the number of data points grows. If there is nothing prior against *f*(*x*), the inference process can begin with an uniformly distributed. *f*(*x*_*i*_|*M*) has an impact on the ultimate distributions *f*(*x*_*i*_|*M*). Monte Carlo techniques must be used to determine or estimate these probability. Equations (3) and (4) show the prior possibility of green and red objects. It is worth noting that, unlike P(C), their probabilities are not modified by measurements. So, if there are any doubts about which *f*(*x*_*i*_|*M*) to choose, one must try them all to assess their systemic influence on the outcomes.

(3) $$\begin{array}{c} P\text{rior Possibility of green}=\frac{\text{Number of green Object s}}{\text{Total Number of Objects}}, \end{array}$$

(4) $$\begin{array}{c} \text{Prior Possibility of red}=\frac{\text{Number of red Objects}}{\text{Total Number of Objects}}. \end{array}$$

A total 50 objects are there. Out of 50 objects, 30 objects are green and 20 are red; our prior possibilities of membership are as shown in.

(5) $$\begin{array}{c} \text{Prior Possibility for green}\propto \frac{30}{50},\\ \text{Prior Possibility for red}\propto \frac{20}{50}. \end{array}$$

After formulating, prior probabilities are categorized in a white circle. Because the objects are highly grouped, it is logical to predict that the more green (or red) items near *N*, the more probable the new cases will be of that hue. To calculate this probability, we create a circle around *N* that contains a number of points (to be determined a priori) regardless of underlying class labels [28]. The number of data points in the circular that belong to each class label is then calculated. We may compute the probability as derived in

(6) $$\begin{array}{c} \text{Probabilities of }N\text{ given green}=\frac{\text{Number of green in terms of }N}{\text{Total Number of green cases}},\\ \text{Probabilities of }N\text{ given red}=\frac{\text{Number of red in terms of N}}{\text{Total Number of red cases}}. \end{array}$$

Because the circle covers three green objects and two red objects, it is evident than chances of *N* provided green is less than chances of *N* given red, thus as applied in

(7) $$\begin{array}{c} \text{Likelihood of }N\text{ given green}=\frac{3}{50},\\ \text{Likelihood of }N\text{ given RED}=\frac{2}{50}. \end{array}$$

Whereas the prior probabilities suggest that *N* belongs to green (due to the fact there are thrice as many green as there are red), the likelihood suggests that *N* belongs to red (because of the fact that there are more red objects in the neighborhood of *N* than green). The overall result in a Bayesian analysis is determined in Equations (8) and (9) integrating both sources of information, namely, the before and the likelihood, to construct a prior distribution using the Bayes' rule [29].

(8) $$\begin{array}{c} \text{Post Probability of }N\text{ being green}\propto \text{Prior Probability of green}\times \text{Likelihood of }N\text{ given green}=\frac{3}{6}\times \frac{3}{50}=\frac{3}{100}, \end{array}$$

(9) $$\begin{array}{c} \text{Post Probability of }N\text{ being red}\propto \text{Prior Probability of red}\times \text{Likelihood of }N\text{ given red}=\frac{2}{6}\times \frac{2}{50}=\frac{2}{150}. \end{array}$$

Therefore, we label *N* as red since it has the highest prior distribution of belonging to that class. Many alternative density measures, such as normally, log-normal type, gamma, and Gaussian, can be used to simulate naive Bayes. Equation (10) is the probability of normal parameters.

(10) $$\begin{array}{c} f\left(x_{i}\left|M\right.\right)=\frac{1}{\sigma_{x}\sqrt{2x}}\exp\left(\frac{{\left(x-\mu_{2}\right)}^{2}}{2\sigma_{x}}\right),-\infty <x<\infty ,-\infty <\mu_{x}<\sigma_{x}>0, \end{array}$$

where *μ*_*x*_ is the mean and *σ*_*x*_ is the standard deviation. Equation (11) is a probability of log-normal type,

(11) $$\begin{array}{c} f\left(x_{i}\left|M\right.\right)=\frac{1}{{x\sigma }_{x}\left(2x\right)\mu^{2}}\exp\left[\frac{\log\left(x{\left(\mu_{x}\right)}^{2}\right)}{2{\sigma_{x}}^{2}}\right],0<x<\infty ,\mu_{x}>0,\sigma_{x}>0, \end{array}$$

where *μ*_*x*_ is the scale parameters, *σ*_*x*_ is the shape parameter, and Equation (12) is the probability of gamma.

(12) $$\begin{array}{c} f\left(x_{i}\left|M\right.\right)=\frac{x/{b_{4}}^{\beta -1}}{b_{4c_{k}}}\exp\left(\frac{-x}{b_{4}}\right)0\leq x<\infty ,b_{4}>0,c_{k}>0, \end{array}$$

where *b*_4_ is a scale parameter and *c*_*k*_ is the shape parameter. Equation (13) is the probability for Gaussian.

(13) $$\begin{array}{c} f\left(x_{i}\left|M\right.\right)=\frac{\beta_{4}\exp\left(\beta_{4}\right)}{x^{4}},0\leq x<\infty ,\beta_{4}>0,x<0>x, \end{array}$$

where *β*_4_ is a mean.

The article "An Image Processing Approach for Detection of Prenatal Heart Disease" was retracted in 2023. Reasons: signs of a paper mill; compromised peer review; unreliable results or conclusions.

### 3.3. Working Principle of Naïve Bayes Classifier

The suggested system's Figure 2 (block diagram off naïve Bayes classifier) illustrates the user collecting the information, the system creating the database (also defined as preprocessing), and the classification algorithm classifying the dataset.

- User: to gather the database, the user is utilized as the input
- System: the document of users are gathered and delivered to the algorithm, which creates the dataset
- Classifier: the predictor is used to estimate whether cardiovascular disease is completely absent, as well as its sharpness, using characteristics such as age, sexual identity, exercise induced angina, breathlessness type, resting blood pressure, resting ECG, serum cholesterol, max heart rate, fasting blood sugar, ST depression induced, number of major vessels, exercise-induced angina, and thalassemia
- Prediction with respect to age: the age of the patients is recorded, and the sickness is evaluated and identified based on their ages
- Analyzing with respect to patient: a specific record is reviewed and sent to the servers, where the outcome is projected based on the patient

### 3.4. Evaluation of Proposed Model

The approach for creating a document classification model starts with data preparation and ends with model assessment. Because certain data are worthless, a preprocessing step has been performed first. The dataset will be more exact as a result. Critical qualities must be chosen after the data preparation step. Crucial in this study refers to how important a characteristic is to the result classes. Classification methods are used to create the model during the classification stage as shown in Figure 3. Therefore, the focus of this research was solely on applying naive Bayes to categorize the papers. Given the probabilistic nature of naive Bayes, the developed naive Bayes classifier wins each basic set by calculating the Bayesian beta value for every dataset. Finally, a collection of the test dataset is used to validate the models. Several assessment metrics (such as accuracy, recollection, and *F*-measure) are used to examine the model's categorization abilities [30]. Moreover, the test reports of naive Bayes would be compared with the results obtained of other classifiers in order to determine whether it is the popular algorithm to utilize.

### 3.5. Data Preprocessing

Several qualities are frequently found to be meaningless. As a result, a stop word removal algorithm was used. A set of stop words has been specified by the humans and hence placed in a text file to initialize the method. The model may then simply match the properties to those preprogrammed stop words. An incomplete data verification algorithm is used after the word removal algorithm. Because data analysis cannot work in the absence of data, this technique is used to locate any incomplete information and assign a rate to it. Originating is the third method used in the preprocessing step. Because some words have similarities but are grammatically distinct (for example, “lender” and “lenders”), as a result, they must be combined into a single characteristic. The texts will have a greater definition (with greater connections) of such terms, as well as the database will be smaller, allowing for quicker processing.

The article "An Image Processing Approach for Detection of Prenatal Heart Disease" was retracted in 2023. Reasons: signs of a paper mill; compromised peer review; unreliable results or conclusions.

### 3.6. Feature Selection

One of the really significant preprocessing procedures in data analysis is feature selection. It is a good image compression approach for getting rid of noise. The main idea behind a feature selection method is to look throughout all possible variations of qualities in the data to determine which group of features is most effective for prediction. As a result, the number of characteristic properties may be decreased, with the most important ones preserved and the superfluous or duplicate ones eliminated and discarded. Throughout this study, many of the publications in the training examples are divided into four groups, by which the model can effectively determine which phrases are often used in each group. Sometimes unnecessary properties can be sorted out this manner. The ideal approach for obtaining a final set of features is to use a subset evaluator; nonetheless, rank searches or random search is recommended for obtaining a solid feature set. As a result, Cfs Subset Evaluator and ranking search are used as the 40 feature selection algorithms in this research. Figure 3 shows the feature that was chosen using the Cfs Subset Evaluator and a ranking evaluation (with gain ratio metric).

### 3.7. Classifier Selection–Document Classification

The number of attributes will be greatly decreased after preprocessing and feature extraction steps, and they will be more exact for use in developing the classifier model. Along with its accessibility and strong performance in documents and text categorization, naive Bayes is chosen as the classifiers in the classification stage, as reported and described. The basic probability classifier is the naive Bayes classifier. A Bayesian classifier's output {*pr*|*cd*} is the likelihood that a source corresponds to category C. Each report contains phrases that are assigned probability depending on the number of times they appear in that text. Using training process, naive Bayes may establish the pattern of evaluating a collection of well-categorized texts and analyzing the information in all classes by creating a list of terms and associated occurrence [31]. As a result, based on highest likelihood function, such a list of word occurrences may be used to categories fresh texts into the appropriate categories.  Figure 4 is the flowchart for naïve Bayes algorithm.

## 4. Experimental Results

The purpose of this assessment is dual. First, it examines if the preprocessing step is beneficial in determining accuracy rate and results in comparison to a case where the dataset has still not been stored and processed. Second, it evaluates the categorization performance in terms of accuracy of several classifiers [32]. The process depends on a dataset of 3000 texts divided into four categories. The documents in the chosen dataset fall into four categories: sports, business, travel, and politics. All four groups are immediately distinguishable. To create the large dataset for the classifiers, 50% of the data (1500 documents) is manually extracted. The remaining 3000 documents are utilized and involved in testing by the proposed classifier. The system is based on the produced naive Bayes classifier, and Table 1 describes the results of applying the naive Bayes classifier to categorize the texts. Surprisingly, the findings of the preprocessed dataset (95 percent) are poorer than those of the unprocessed dataset (97 percent). As a result, in order to attain a better outcome, the preprocessed model must be adjusted. Because the preprocessing step is used in all cases, the adjustments are applied during the feature selection stage. The feature selection is made using the Cfs Subset Evaluator and rank searching (using the gain ratio measure). As a result, a different method of rank inquiry has been tested. This time, 89 characteristics were chosen using the Chi-square feature selection algorithm. Rather of the 75 qualities that were previously picked, 89 attributes were entered this time. After employing the Chi-square classification algorithm, the outcome has improved. The accuracy has increased by 0.1 percent. Although the difference is minor, preprocessing and feature selections have been shown to help achieve higher classification results. Another important fact is that even the time it takes to create the image has improved dramatically that after set of attributes has been lowered from 9.6 secs to roughly 0.19 secs.

The article "An Image Processing Approach for Detection of Prenatal Heart Disease" was retracted in 2023. Reasons: signs of a paper mill; compromised peer review; unreliable results or conclusions.

### 4.1. Model Evaluation

80 percent of the total of the database is utilized to test and validate the model. The collected cases are then used as a benchmarks sample for machine learning algorithms. System capacity may be measured in terms of recall, accuracy, and *F*-measure by evaluating the current class of the occurrence with the expected by the classification model. The outcomes of not preprocessing and preprocessing are combined to further assess the effectiveness of the suggested preprocessing stage. But if the outcomes are even worse than since no preprocessing is done, then parameters must be adjusted and fine-tuned. As a result, the model must be rebuilt. This procedure will be repeated until a satisfactory categorization result is achieved [33]. Moreover, the naive Bayes classifier would be compared to certain other classifications (such as DT, NN, and SVM) to see if it is the highest among them. Equations (14)–(17) formulate the parameters such as accuracy, recall, precision, and *F*-measure.

#### 4.1.1. Accuracy

Accuracy is defined as the product of sensitivity and prevalence multiplied by the product of specificity. Accuracy comparison of three parameters such as recall, precision, and *F*-measure on both with preprocessing and without preprocessing and feature extraction is as shown in Table 1.

(14) $$\begin{array}{c} \text{Accuracy}=\left(\text{Sensitivity}\right)\left(\text{Prevalence}\right)+\left(\text{Specificity}\right)\left(1-\text{Prevalence}\right). \end{array}$$

#### 4.1.2. Recall

The recall is a measurement of how well our model detects true positive aspects. As a result, recall informs us how many patients we accurately recognized as having heart disease out of all patients.

(15) $$\begin{array}{c} \text{Recall}=\frac{\text{Number of relevant documents retrieved}}{\text{Total Number of relevant documents}}. \end{array}$$

#### 4.1.3. Precision

Precision is one measure of a machine learning techniques, and the accuracy of a model's rates will increase. The proportion of true positives based on number of predictions made is known as precision.

(16) $$\begin{array}{c} \text{Precision}=\frac{\text{Number of documets relevant for prediction}}{\text{Total Number of relevant documents}}. \end{array}$$

#### 4.1.4. *F*-Measure

*F*beta-measure is a fixed metric that may be used to evaluate a binary classifier that refers to positive that have this. Precision and recall are used to construct the *F*beta-measure. Precision is a statistic for determining the percentage of true positive class predictions.

(17) $$\begin{array}{c} F–\text{Measure}=\frac{2\times \text{Rebuilt}\times \text{Prediction}}{\text{Recall}+\text{Precision}}. \end{array}$$

Following a discussion on the significance of data preparation and feature selection, the next experiment will determine whether naive Bayes is the better model among the others. Three distinct classifications were used for screening in order to achieve this goal. SVM (the “SMO” function in WEKA), NN (the sluggish “IBk”), and DT (the branch “J48”) are the classifiers. The preprocessed datasets (with 90 characteristics) are utilized to evaluate this research. With precision, recall, and *F*-measure, Table 2 summarized all of the accuracy data. The accuracy score of naive Bayes is the highest along with other classifiers, as indicated in the table.

In the coronary heart dataset, there are a maximum of 570 records. The entire records are partitioned into two large datasets, including one training and another one for testing. The training process has 300 records and the checking dataset contains 275 data. For the research, the data mining program MATLAB is employed. Originally, the dataset comprised several variables in which there was no value in the entries. The replacement incomplete values filtering in MATLAB was used to find all these replace them with the most relevant values. The replace missed values filter searches all entries and uses the mean mode approach to replace the lost values. Preprocessing stage is the term for this procedure. Different data mining algorithms such as neural networks, *K*-nearest neighbor, random forest, naive Bayes classifier, and decision trees were used following preprocessing the dataset. The rate of accuracy using training and testing data in various machine learning technique is mentioned on Table 3. To measure the classification performance, a confused matrix is formed. The number of instances allocated to each class is shown in a contingency table. Researchers had two classes in our study with 2 × 2 matrix.

The article "An Image Processing Approach for Detection of Prenatal Heart Disease" was retracted in 2023. Reasons: signs of a paper mill; compromised peer review; unreliable results or conclusions.

The goal of this study is to determine if a patient may suffer heart problems. On the datasets, this study focused on trained data mining and machine learning approaches such as naive Bayes, random forests, decision trees, and *K*-nearest neighbor. The WEKA tool was used to conduct a number of tests involving various classifier algorithms. The research was conducted on an Intel Corei7 8th generations processor with a clock speed of up to 4.1 GHz and 8 GB of RAM. A training data and a test set were created from the database. To obtain an average accuracy, the data is preprocessed and monitored clustering algorithms such as naive Bayes, *K*-nearest neighbor, random forest, and decision trees are used. The percentage of accuracy is estimated for various classifiers using python programming with training and testing data as shown in Table 3. Using this prediction naïve Bayes classifier has achieved good accuracy compared with other techniques.

The naive Bayes classifier has an accurateness of 98% and a recall value of 99.7% when using the random resampling strategy. The KNN and decision tree methods also result in positive outcomes. Accuracy performance of various classifiers are shown in Figure 5. In all sampling techniques, this strategy provides better accuracy. This procedure, however, is not dependent on any optimization approach.

#### 4.1.5. Specificity

The technique of measuring the accurate classification of nondiseased patients to the total nondiseased patients is known as specificity. Specificity comparison of various classifiers is mentioned in Table 4, and the formulated part of specificity is derived in Equation (18).

(18) $$\begin{array}{c} \text{Specificity}=\frac{\text{True non}‐\text{diseased patients}}{\text{Total non}‐\text{diseased patients}}\times 100. \end{array}$$

Naive Bayes classifier yields the best specificity. The best specificity is reached by the NB classifier, according to the experimental results. All classifiers are subjected to 2 × 2 matrix validation. Table 4 summarizes the efficiency of these classification based on the foregoing findings; the suggested system is capable of detecting and classifying heart diseases.  Figure 6 shows a graphical representation of this outcome comparison for specificity.

The article "An Image Processing Approach for Detection of Prenatal Heart Disease" was retracted in 2023. Reasons: signs of a paper mill; compromised peer review; unreliable results or conclusions.

#### 4.1.6. Sensitivity

The technique of measuring the total number of diseases to the correct classification of diseased people is known as sensitivity. Sensitivity comparison of various classifiers is mentioned in Table 4, and the sensitivity calculation is denoted in Equation (19).

(19) $$\begin{array}{c} \text{Sensitivity}=\frac{\text{True diseased people}}{\text{Total diseased people}}\times 100, \end{array}$$

After analysis, NB yields better sensitivity. The best sensitivity is reached by the NB classifier, according to the experimental results. All classifiers are subjected to 2 × 2 matrix validation. Table 4 summarizes the performance of these classifiers. Based on the foregoing findings, the suggested system is capable of detecting and classifying prenatal heart diseases.  Figure 7 shows a graphical representation of this outcome comparison for sensitivity.

The purpose of this research is to appropriately classify the input experimental information into four different categories (business, sport, politics, and travel). To begin, it provided 2000 documents for every category as a database for building the classifier model. To create and validate the classifier model, the whole 3000 papers will be divided into two databases, namely, the training phase and the testing set, with 40% of the documents going to the training set and 60% going to the testing set. These documents have already been preprocessed into 1320 characteristics (in terms of mathematical values) and 1 resolution attribute in their representations (in term of nominal values). Figures 5–7 shows the classification of specificity, sensitivity, and accuracy. There are no variables with missing information, and all numeric properties are defined using the word intensity document frequencies (TFIDF).

## 5. Discussion

The naive Bayes classifier is unexpectedly effective in practice, despite its unreasonable posterior probability, because its classification choice is typically accurate even though its probability estimations are incorrect. Although several naive Bayes optimization requirements have been found in the prior, a better knowledge of the data properties that influence naive Bayes effectiveness is still needed. Our overarching goal is to comprehend the data qualities that influence naive Bayes effectiveness. Our method employs numerical simulations, which allow for a thorough examination of categorization accuracy for a variety of completely random issues. We investigate the effect of distributed volatility on classification algorithm, demonstrating that only certain almost deterministic, or reduced, relationships result in good naive Bayes results. We show that naive Bayes is most effective in two situations: entirely independent variables (as expected) and operationally dependent elements (which is surprising). Between such two extreme values, naive Bayes has provided best performance. Unexpectedly, the amount of feature interdependence assessed as the category similarity measure between both the features has no clear correlation with the efficiency of naive Bayes [34]. However, the leakage that attributes provide well about category when using a naïve Bayes model is a stronger predictor of reliability. To find out the correlation between such calculated by using following and the behavior of naive Bayes, more empirical and conceptual research is needed. Analyzing naive Bayes on real applications of almost dependency, describing other domains of naive Bayes optimization problem, and researching the impacts of multiple integral feature on the naïve Bayes classification error rate are some of the other directions. Finally, a good comprehension of the effect of the apparent inconsistency on categorization can be used to develop better concerned with methods for learning effective Bayesian classifier and probability-based inference, such as method to resolve the issue assigned tasks, using naïve Bayes classifiers.

The article "An Image Processing Approach for Detection of Prenatal Heart Disease" was retracted in 2023. Reasons: signs of a paper mill; compromised peer review; unreliable results or conclusions.

## 6. Conclusion

The main goal is to establish several data mining approaches that can be used to accurately forecast cardiac disease. Our goal is to provide efficient and reliable predicting with a smaller number of features and tests. Only 14 critical features are considered in this study. Naive Bayes, *K*-nearest neighbor, random forest, and decision tree were the four data mining categorization algorithms I used. The information was preprocessed before being utilized in the algorithm. The techniques with the greatest outcomes in this model are naïve Bayes classifier, and the after constructing four algorithms are KNN and decision tree. Case of study discovered that naïve Bayes classifier had the best accuracy. Additional data mining methods, such as time series data, segmentation and connection rules, evolutionary algorithms, and support vector machine can be used to enhance this research. Given the findings of this research, more complicated and combined models are needed to achieve better accuracy in the early detection of heart disease. In this research, researchers propose using a multimodal maximum possible series data pattern with a naive Bayes classifier to classify electrocardiogram abnormalities in the lack of actual knowledge. It also outperforms methodological approaches with a reliability rate of 97 percent and a precision rate of 94 percent.

## Figures and Tables

**Figure 1:** Proposed model for machine learning.

**Figure 2:** Block diagram of naïve Bayes classifier.

**Figure 3:** Proposed naïve Bayes algorithm.

**Figure 4:** Flowchart of naïve Bayes classifier.

**Figure 5:** Accuracy comparison of various classifiers.

**Figure 6:** Specificity comparison of various classifiers.

**Figure 7:** Sensitivity comparison of various classifiers.

**Table 1:** Accuracy rate of naïve Bayes classifier using without processing and feature extraction and with processing and feature extraction.

Preprocessing	Instance classified in correct format	Instance classified in incorrect format	Recall	Precision	*F*beta-measure
Without processing and feature extraction	2711	88	0.97	0.95	0.97
With processing and feature extraction	2654	125	0.96	0.94	0.96

**Table 2:** Accuracy rate of naïve Bayes classifier using various features and dataset.

Preprocessing	Instance classified in correct format	Instance classified in incorrect format	Time (secs)	Recall	Precision	*F*beta-measure
Feature extraction without preprocessing	2711	86	9.6	0.97	0.97	0,95
Feature extraction–gain ratio with preprocessing	2535	121	0.15	0.96	0.95	0.94
Feature extraction-chi-square with preprocessing	2610	84	0.2	0.98	0.96	0.98

**Table 3:** Accuracy comparison using training and testing data with various techniques.

Accuracy	NBC	DT	RF	KNN
Training dataset	89.15	78.3	74.6	84.3
Testing dataset	90.5	83.5	78.9	82.94

**Table 4:** Comparison of accuracy, specificity, and sensitivity using various techniques.

Methods	NBC (%)	KNN (%)	DT (%)	RF (%)
Accuracy	97	92	89	79
Specificity	96	88	78	75
Sensitivity	94	87	74	72

## Data Availability

The data used to support the findings of this study are included within the article. Further data or information is available from the corresponding author upon request.
